# The Application of Biomechanics Combined with Human Body Structure in Volleyball Technical Analysis

**DOI:** 10.1155/2022/5287538

**Published:** 2022-05-18

**Authors:** Wei Jiang, Kai Zhao

**Affiliations:** China Volleyball College, Beijing Sport University, Beijing 100089, China

## Abstract

With the development of volleyball, the development of traditional school volleyball has been paid increasing attention. This has also aroused the concern of schools, coaches, and athletes and has become the focus of volleyball development and reserve talent training. The purpose of this paper is to use the knowledge of biomechanics to study serving technology and attacking technology in volleyball. In the aspect of biomechanics, this paper proposes the finite element modeling theory of the human body. The upper limbs of volleyball players are modeled and analyzed, and four powerful teams are selected for video analysis of volleyball offensive skills. The overall difference between athletes in different groups is very obvious. The phase with the longest time and the greatest difference was the P3 phase, which took 0.802 ± 0.085 seconds.

## 1. Introduction

In 2018, air volleyball appeared in the 14th Gansu Provincial Games as an official event. This is not only because air volleyball is simpler than hard volleyball, but it also weakens the rigid requirements for physical fitness and pays more attention to the use of technology and tactics. The number of people participating is large. And it is also in line with the theoretical thought of “widely carrying out national fitness activities and accelerating the construction of a strong sports country” put forward by the General Secretary in the report of the 19th National Congress of the Communist Party of China.

However, there are a series of problems in the development of traditional project schools at present: the contradiction between the training and learning of the students participating in the training; the lack of special coaches and unscientific training; the coaches have to take classes and bring training, the work pressure is high, the salary is meager or even no, which leads to the lack of enthusiasm of the coaches and the decline of the quality; the athletes have few opportunities to participate in the competition, and the students are not willing to spend a lot of energy on practice; talent delivery channels are relatively narrow and limited. Most parents worry that their children will not have excellent sports performance and will delay cultural learning, so they pay more attention to their children's intellectual development and cultural knowledge learning; areas with good economic conditions develop better, and areas with poor economic conditions are difficult to develop. Therefore, how to carry out scientific management and effective training in traditional project schools to ensure the comprehensive and harmonious development of students' morality, intelligence, physique, and beauty is an important issue faced by school sports and competitive sports workers.

The biomechanical volleyball project has the following two innovations: (1) With the rapid development of air volleyball today, the requirements for attacking technology are getting higher and higher. For a mature team, a strong offense is a key to winning games. Therefore, this paper takes air volleyball players as the analysis object. (2) This paper conducts data statistics and analysis on the video playback of the men's top four teams in the 14th game. It takes the offensive technical effects of the top four teams as the starting point, analyzes the advantages and disadvantages of each team in various offensive technologies, and draws the key to victory for each team. This provides a reference for the faster and better development of air volleyball.

## 2. Related Work

At present, it is the golden period for the development of air volleyball. By consulting a large number of works of literature on the development of gas volleyball, it is found that the current development of this sport in the southern region is better than that in the northern region. The biomechanics of the eye were analyzed by Kling and Hafezi. They argue that corneal shape is a determinant of eye refraction but itself is determined by its biomechanical properties [1]. Gajewski et al. conducted an experimental study on 100 young athletes to determine the determinants of maximal strength during vertical jumping and to elucidate the relationship between jump height and the ability to exert maximal strength. The models were built using multiple regression analysis and allometric scaling. Their model is used to calculate the expected power value of each participant, which is closely related to the actual value [2]. Baleen whales were studied by Goldbogen et al.. They reviewed the current state of the field by exploring several hypotheses aimed at explaining how baleen whales feed. Despite significant progress, significant questions remain about the processes behind these extreme feeding mechanisms. These mechanisms enabled the evolution of the largest animals ever created [3]. Guerra et al. describe a class of nonlinear observers based on the state-space descriptor form and the Takagi-Sugeno model. Convergence conditions for prediction errors are investigated through an LMI-based design. Finally, its application in human standing biomechanics is presented. The unknown input observer is designed to calculate the joint torque and velocity from position video-based measurements [4]. Chang et al. present a study on the relationship between neutrophil proteases and protease inhibitors in premature infants with chronic lung disease (CLD). They measured various factors, including neutrophil elastase (NE) activity, cell counts, and metalloproteinase (MMP)-9. The results showed that MMP-9 and NE activity affected CLD development with increasing protease and inhibitor concentrations [5]. The cellular mechanisms in human biomechanics were investigated by Chang and Su. Their experimental results suggest that heme-induced heme oxygenase may be a general response to oxidative stress by increasing bilirubin and ferritin levels. It can thus provide a major cellular defense mechanism against oxidative damage [6]. However, after related research, it can be found that although the research on biomechanics is very deep, the biomechanical analysis of volleyball is less, and more volleyball skills are updated and upgraded through video analysis.

## 3. Volleyball and Biomechanics

### 3.1. Volleyball Events

Air volleyball is a new type of sport that was first born out of hard volleyball in China. Its advent enriched the world volleyball system [7, 8]. Because air volleyball has a good fitness effect and entertainment value, it also has a certain technicality, which is in line with the guiding ideology of “health first” proposed by China and is suitable for people of different ages to learn. Therefore, since its inception, it has been extremely popular and has swept the country. In 1989, the state established a promotion group dedicated to the promotion of air volleyball and proposed to promote the development and popularization of air volleyball across the country. At the same time, it is also required to develop air volleyball as a national fitness sport, and it is proposed to focus on the development of factories, enterprises, and school communities [9]. For example, the middle-aged and elderly air volleyball series championships held across the country have made increasingly people understand the sport and promote its development. As shown in Figure 1.

#### 3.1.1. Air Volleyball

Air volleyball is a local mass entertainment and fitness activity born and raised in China. In 1984, to enrich the daily life of retired employees, the Jining Branch of the Hohhot Railway Bureau allowed retired and retired employees to play with balloons on the volleyball court without any rules for entertainment [10, 11]. However, balloons are not heavy enough and explode easily. Therefore, the employees invented a way to put two balloons together and later replaced them with soft plastic balls for children to play with. With the continuous development of the sport, simple rules of the game were drawn up with reference to the rules of 6-a-side volleyball, and this activity was named “air volleyball.”

#### 3.1.2. Volleyball Technique

Volleyball technique refers to the general term that players can use a variety of reasonable hitting actions and other coordinated actions to complete the game within the scope allowed by the rules.

Volleyball offensive technique specifically refers to the organized, purposeful, and legal means used by the players of both participating sides to make the volleyball fall on the opponent's court or make the opponent make mistakes and win the score during the game.

The offensive effect refers to the result obtained after the offensive behavior occurs, and the quality of the offensive effect is one of the important indicators to test the offensive.

### 3.2. Development of Volleyball Projects-Taking Kunming, Chengdu as an Example

#### 3.2.1. In terms of Coaches

The age structure of after-school training coaches in traditional volleyball projects is basically reasonable, forming a combination of old, middle, and light. 50% of Chengdu is mainly young and middle-aged backbone teachers aged 36–50. The coaches in Kunming are mainly under the age of 35. Relatively speaking, Chengdu coaches are more energetic. The economy and external factors are relatively stable, and the social practice experience is rich. In terms of training and competition, it is more dominant than Kunming. The coaching years of the coach are basically the same as the coach's age. Chengdu coaches are mainly 6–10 years old, accounting for 31.2%. Kunming coaches are mainly concentrated in 1–5 years, accounting for 50%. The coaches in the two cities have short years of coaching, and it is necessary to strengthen the training and learning of the coaches. However, the job training of coaches in the two cities is not perfect, has not been fully implemented, and has not achieved practical results. The coaches in the two cities mainly have bachelor's degrees as the main force, and there are very few master's degrees. Therefore, it is necessary to inject more highly educated talents to drive the development of scientific research and promote the development and popularization of volleyball. In terms of professional titles, Kunming is mainly junior and senior, accounting for 40% and 30%, respectively. Chengdu coaches are mainly senior, accounting for 40.6%, followed by super and junior. This shows that the coaches of the two cities are generally excellent old coaches combined with new coaches, which is conducive to the development of school volleyball after-school training and the improvement of training level year by year. To improve the technical and tactical training capability and adapt to the fast-paced competitive competition, it is necessary to combine theory with practice and utilize existing resources. In training practice, problems are constantly found and research solutions are sought, and the characteristics and rules of techniques and tactics can be explored to find the most effective training methods and improve the efficiency of athletes' training [12, 13]. In terms of extracurricular training, the coaches in the two cities mainly simply formulate weekly and stage training plans and lack detailed and thorough training plans during class hours. Through surveys and statistics, it is found that coaches in Chengdu are more serious about writing training plans than those in Kunming. However, coaches in both cities usually have a double duty. They have to complete the daily gym class and lead the training team in their spare time. In addition, many school coaches are responsible for both junior high school and high school training and athletes' registration for competition, registration, and athlete level approval, all of which need to be undertaken by the coaches. Coaches have a lot of work and spend a lot of their energy and spare time, but the gains are not positively related to their efforts.

In particular, the average subsidy of 300 yuan per month for coaches in Kunming is 5–10 yuan per training, which is similar to unpaid labor. And the subsidy of 300 yuan is related to the performance of the game. If the performance of the game is not good, part of it will be deducted. In the year-end performance appraisal, only 1 point can be added to the total score, which cannot be proportional to the hard work and time spent. It has no effect on the professional title, which creates a sense of unfairness to the coach and seriously dampens the coach's enthusiasm. This is also one of the important factors affecting the level of volleyball in Kunming. Therefore, it should be given high priority. 50% of the coaches of the Chengdu Volleyball Traditional School are basically satisfied with the treatment of leading team training, 31.5% are relatively satisfied, and the satisfaction level with the volleyball team training allowance is over 80%. Among the five schools surveyed, three of them spent 70–100 yuan per training. If you achieve excellent results in the competition, the coach can be rewarded 1000–5000 yuan according to the competition level and situation. It can be clearly seen that there are significant differences in the treatment of coaches in the two cities. From the overall point of view of the coaches of the after-school training team, Chengdu is more favorable than Kunming, and the coaches are more motivated, which is more conducive to promoting the development of volleyball [14].

#### 3.2.2. Athletes

Comparing the traditional volleyball schools in Chengdu and Kunming, among the athletes who participated in volleyball after school training, 60.4% of the athletes in Chengdu were very interested in volleyball training, and 44.9% of the athletes in Kunming were very interested. This is good data. Because people are willing to pay for things they are interested in, and they can enjoy it no matter how hard or tired they are. However, the short time to participate in volleyball shows a “lag.” Chengdu athletes start volleyball training at the age of 11–12 on average. Most of the athletes in the traditional sports school for volleyball in Kunming start volleyball training at the age of 13–15. Athletes train for a relatively short period of time. Most athletes are exposed to volleyball training during junior high school. In addition, this paper also conducts a T on the training years and sports grades of athletes in the two cities. The independent sample *T*-test result of athletes participating in training in the two cities was *T* = −0.12 (*p* < 0.01). There are obvious differences in training years between traditional volleyball players in Chengdu and traditional school players in Kunming. The independent sample *T*-test for the athletes' sports grades in the two cities was *T* = 3.25 (*p* < 0.01), indicating that there were significant differences in the sports grades of the two cities. Therefore, it can be seen that the average sports years of athletes in Chengdu are longer than those in Kunming, and the sports level is also significantly higher than that in Kunming. In terms of daily training, the athletes of the two cities follow the coaches' arrangement and train with the school's after-school training team for a long time, while the training time in Kunming cannot be guaranteed. Due to site constraints and various factors, training is usually arranged at 12:50–13:50 or 5:50–6:50 noon, and normal training is often not possible due to bad weather, such as rain and snow. Therefore, from the perspective of athletes, athletes from traditional schools in Chengdu have more advantages than those in Kunming.

#### 3.2.3. Athlete Selection and Transportation

The most concerned about the selection of coaches in the two cities is the physical shape and physical quality, followed by the coaches' own experience. However, there are a few aspects of bone age, coordination, personality, and psychological factors, indicating that the selection of materials is not perfect. The source of traditional volleyball projects in Kunming City mainly relies on the annual registration examination for the selection of schools for special student resources. Only 10% of the students are trained by their own schools. 80% of the students in the traditional school of volleyball in Chengdu come from the lower schools of the school. The outstanding students can be directly promoted to the higher school of the school, and then the special enrollment examination will be adopted to select the best. In terms of athlete delivery, athletes who are carefully cultivated by coaches are lost due to further education or graduation [15, 16]. There is a lack of drastic measures for athletes to have excellent results. In addition, the continuous development of students with specialties cannot be guaranteed, which is also one of the factors affecting the development of platoons.

#### 3.2.4. Competition Aspects

The coaches reported that the competition system in the province is not in line with the development of national and even world volleyball, and athletes have few opportunities to participate in the competition. In the volleyball events of the two cities, the common situation of the traditional school competition is the annual provincial traditional school competition and the provincial youth championship. However, not all schools participate every time. Some schools have not participated in provincial competitions for several years and are not eligible to participate in national competitions. In general, athletes lack a competition platform and lack of competition experience. In the official competition, the daily training level cannot be played normally, resulting in unsatisfactory competition results. As a result, a phenomenon is formed. The higher the sports level, the more opportunities to participate in the competition, and the faster the athlete's technical level will improve. However, schools with poor technology have fewer opportunities for exercise and less financial support from the government and schools, which makes the development of sports levels slow. After-school training teams from the two cities have few traditional schools participating in national-level competitions. Among them, only Chengdu Northwest Middle School and Chengdu No. 7 Middle School participated in the National U18 Youth Championship and won the 9th and 11th, respectively; no school in Kunming has participated in the national competition. This shows that the technical level of volleyball in traditional schools in the two cities is not excellent enough [17].

### 3.3. Training Conditions and Guarantees

The traditional volleyball school venues in Chengdu can basically meet the needs of after-school training, but there are also schools with insufficient venues; there is a big gap in the venues and facilities of the traditional volleyball schools in Kunming; the funding problem has seriously restricted the development of volleyball in Kunming. There is a sense of helplessness among coaches raising funds during the survey. To ensure daily training and competition, the coaches can only compress the usual expenses and collect training fees from the students. Solving the funding problem of the traditional volleyball school in Kunming is the top priority. In terms of capital investment in Chengdu, there are corresponding incentive policies to stimulate the interest of coaches and athletes. However, in terms of capital investment in Chengdu, there is a trend of “cutting down the weak to support the excellent.” Excellent schools have more support and incentives, and schools are unfavorable in the initial stage, resulting in slower development.

### 3.4. Theoretical Basis of Human Body Finite Element Modeling

#### 3.4.1. Common Unit Types of Human Tissue

The element types commonly used in the modeling of human biomechanical finite element models include shell elements, tetrahedral elements, and hexahedral elements. Among them, shell elements are often used to simulate thin film tissues such as skin and blood vessels. For important solid tissues such as bone and muscle, tetrahedral or hexahedral solid elements are often used to simulate [18, 19].

Tetrahedral elements are the simplest and most commonly used type of solid element. Each tetrahedral element has 4 nodes, and each node has 3 degrees of freedom, as shown in Figure 2. Its displacement formula and shape function matrix are shown in the following formulas.


(1) $$\begin{array}{c} u\left(x,y,z\right)=a_{0}+a_{1}x+a_{2}y+a_{3}z,\\ v\left(x,y,z\right)=b_{0}+b_{1}x+b_{2}y+b_{3}z,\\ w\left(x,y,z\right)=c_{0}+c_{1}x+c_{2}y+c_{3}z,\\ u{\left(x,y,z\right)}_{3\times 1}=\left[\begin{array}{c} u\\ v\\ w \end{array}\right]=N_{3\times 12}\cdot q_{12\times 1}^{e}. \end{array}$$

Among them, the function matrix can also be expressed as follows:

(2) $$\begin{array}{c} \left[\begin{array}{c} u\\ v\\ w \end{array}\right]=\left[\begin{array}{ccccccc} N_{1} & 0 & 0 & \cdots & N_{4} & 0 & 0\\ 0 & N_{1} & 0 & \cdots & 0 & N_{4} & 0\\ 0 & 0 & N_{1} & \cdots & 0 & 0 & N_{4} \end{array}\right]\cdot q_{12\times 1}^{e}. \end{array}$$

In the formula,

(3) $$\begin{array}{c} N_{i}=\frac{1}{6V\left(a_{i}+b_{i}x+c_{i}y+d_{i}z\right)},\\ q_{12\times 1}^{e}=\left[\begin{array}{ccccccc} u1 & v1 & w1 & \cdots & u4 & v4 & w4 \end{array}\right]. \end{array}$$

*V* represents the volume of the tetrahedral element, and *a*_*i*_, *b*_*i*_, *c*_*i*_, and *d*_*i*_ are constants. Therefore, the shape function matrix is a constant strain matrix. That is, the tetrahedral element is a constant strain element.

The hexahedral element has 8 nodes, each with 3 degrees of freedom. The hexahedral element, therefore, contains a total of 24 degrees of freedom, as shown in Figure 3. Its displacement formula and shape function matrix are shown in the following formulas:


(4) $$\begin{array}{c} u\left(x,y,z\right)=a_{0}+a_{1}x+a_{2}y+a_{3}z+a_{4}xy+a_{5}xz+a_{6}yz+a_{7}xyz,\\ w\left(x,y,z\right)=b_{0}+b_{1}x+b_{2}y+b_{3}z+b_{4}xy+b_{5}xz+b_{6}yz+b_{7}xyz,\\ v\left(x,y,z\right)=c_{0}+c_{1}x+c_{2}y+c_{3}z+c_{4}xy+c_{5}xz+c_{6}yz+c_{7}xyz,\\ u{\left(x,y,z\right)}_{3\times 1}=\left[\begin{array}{c} u\\ v\\ w \end{array}\right]=N_{24\times 1}\cdot q_{24\times 1}^{e}. \end{array}$$

It can be seen from the above formula that the displacement of the hexahedral element is a linear displacement. The displacement of the common nodes of two adjacent elements on the boundary is continuous, which is more accurate than that of tetrahedral elements. Therefore, the lower limb model is mainly modeled with hexahedral elements.

Kalman filter is an efficient recursive filter. Extended Kalman filter utilizes the local linearity of nonlinear systems to achieve the optimal estimation of body pose through continuous iteration. Due to the advantages of smoother attitude angle and less noise disturbance calculated by this method, this method is used for signal processing of inertial navigation system in this study. That is, Kalman filtering is used to fuse the triaxial acceleration, triaxial angular velocity, and triaxial gyroscope data. Thereby, the gliding speed, body position, and body posture of the athlete can be obtained. The data are then fused using an extended Kalman filter to obtain the corresponding parameter information after calibration.

Extended Kalman filter system model:

(5) $$\begin{array}{c} \dot{x}\left(t\right)=f\left(x\left(t\right),t\right)+g\left(x\left(t\right),t\right)w\left(t\right),w\left(t\right)∼N\left[0,Q\left(t\right)\right]. \end{array}$$

Measurement model:

(6) $$\begin{array}{c} z\left(t\right)=C\left(x\left(t\right),t\right)+v\left(t\right),v\left(t\right)∼N\left[0,R\left(t\right)\right]. \end{array}$$

Initial conditions:

(7) $$\begin{array}{c} x\left(t\right)∼N\left({\hat{x}}_{0},P_{0}\right),\\ \text{Cov}\left[w\left(t\right),v\left(\tau \right)\right]=0. \end{array}$$

State estimation formula:

(8) $$\begin{array}{c} x\left(t\right)=F\left(\hat{x}\left(t\right),t\right)+K\left(t\right)\left[z\left(t\right)-C\left(\hat{x}\left(t\right),t\right)\right]. \end{array}$$

Error covariance:

(9) $$\begin{array}{c} \dot{p}\left(t\right)=F\left(\hat{x}\left(t\right),t\right)p\left(t\right)+p\left(t\right)F^{T}\left(\hat{x}\left(t\right),t\right)+G\left(t\right)Q\left(t\right)G^{T}\left(t\right)-K\left(t\right)R\left(t\right)K^{T}\left(t\right). \end{array}$$

Gain matrix:

(10) $$\begin{array}{c} K\left(t\right)=P\left(t\right)H^{T}\left(\hat{x}\left(t\right),t\right)R^{-1}\left(t\right). \end{array}$$

#### 3.4.2. Commonly used material models of human tissue

Human tissue can be divided into two categories, hard tissue and soft tissue. The hard tissues are mainly human bones, while the soft tissues include brain tissue, internal organs, muscles, ligaments, and cartilage [20]. Among them, the bones are usually simulated by elastic-plastic materials, and this model can more realistically reflect the material properties of human bone. When the bones are divided by shell elements, the material model is mostly piecewise linear elastic-plastic material. When using solid element division, exponentially hardening elastoplastic material simulation is often used. Its stress-strain relationship has the following exponential law:

(11) $$\begin{array}{c} \sigma =a+b\varepsilon_{p}^{n}. \end{array}$$

In the formula, *σ* represents the true stress of the tissue. *a* represents the initial yield stress. *ε*_*p*_^*n*^ stands for effective plastic stress. *n* represents the hardening index. *b* represents the correspondence coefficient, and the effect of strain rate is considered by the Cowper-Symonds method.

The biological soft tissue is mostly simulated by elastic or viscoelastic materials. Among them, skin, cartilage, etc. are usually simulated by elastic materials, while brain tissue, internal organs, muscles, etc. have obvious viscoelastic characteristics, so viscoelastic material models are used. Its shear elastic model is given by the following:

(12) $$\begin{array}{c} G\left(t\right)=G_{\infty }+\left(G_{0}-G_{\infty }\right)e^{-\beta }t. \end{array}$$

In the formula, *G*_*∞*_ is the long-term shear modulus, *G*_0_ is the short-term shear modulus, and *β* is the decay coefficient.

## 4. Volleyball Biomechanical Analysis

### 4.1. The Objects of Research

Among the junior students of a sports college majoring in volleyball, 8 athletes with better serving skills in the game were selected as the test subjects. These athletes have been trained for a long time and have performed well in previous competitions. They can more proficiently complete the serving action and can meet the relevant requirements of this work action analysis. All test subjects only performed low-intensity daily training and did not arrange any other amount of exercise in the 24 hours before the study. To maintain a stable mood, a sufficient warm-up exercise is required for this work so that they can play their respective levels stably. To avoid interfering with the test results due to gender differences, all 8 athletes were selected males. In addition to analyzing the relevant characteristics of the overall motion structure of the 8 test subjects' serving actions, this paper will also divide the test subjects into two groups, the ordinary group and the excellent group, according to the two factors of the test players' grade and the coach's evaluation. The related technical movement characteristics of the above two groups of athletes were compared and analyzed. The details of the basic information of the tested athletes are shown in Table 1.

### 4.2. Methods of Research

In this paper, the biomechanical analysis of volleyball serving technology is carried out by using five research methods: literature method, image measurement method, expert interview method, experimental method, and mathematical statistics method. By consulting the literature and processing them, the research design and conception of this thesis have been provided as a reference. Materials for further study and analysis are provided by image metrology. The feasibility and innovation points of the research are clarified through the expert antitalk method, which provides directional guidance for the key points of the research. The relevant kinematic parameters were measured experimentally to provide reliable data for the overall study. The original data is counted and processed by the mathematical statistics method, and the correlation analysis is carried out on the factors that may affect the performance of the server action, which provides the basis for the research conclusion of this paper [21, 22]. The schematic diagram of the technical route is shown in Figure 4.

Through the high-speed camera method, the serve technique is analyzed in many ways. Only in this way can we determine the key points of the kinematic factors of each stage of the batting action technique and the corresponding displacement, speed, trajectory, and time node distribution of each link in the use of the batting technique, as well as the relationship between each stage. Among them, the image test process is as follows.

The movements of the subjects will be video recorded using 2 high-speed video recording machines. One of them is fixedly installed on the left side of the subject, with a distance of 5 m from its front, and the installed tripod is 1.1 m high. The other one is installed on the left front of the subject, keeping a distance of 5 m from each other, and the installed tripod is 1.1 m high. The included angle between the main optical axes of the two devices is 60 degrees (as shown in Figure 5). The lens orientation is perpendicular to the moving surface. Before filming, signs with reflective functions are pasted on each joint point of the subject to effectively facilitate subsequent work and reduce test errors. At the same time, the sidekicks of each subject were recorded and related image information was obtained. APAS was used to find the shear motion signal of the sync point. Digital processing is then enhanced to obtain the final information for research.

### 4.3. Division of Research Stages

To better analyze the characteristics of the batting action, excluding the stage action of returning the leg to the actual combat position after the kick is not within the scope of this study. The batting action is divided into 3 action stages and 4 action moments. In this way, a clearer and more thorough understanding of the important stages of the sidekick technical action can be obtained. The process is shown in Figure 6.

The first stage starts from preparing to serve and ends when the ball leaves the hand. The second stage is from the moment the ball leaves the hand to the time it falls back into the hand. The third stage is from the ball in hand to the end of the serve. The specific process and content of the three action stages and four action stages are shown in Table 2.

### 4.4. The Overall Movement Structure and Characteristics of the Tested Athletes

#### 4.4.1. Time-Varying Characteristics

It can be seen from Figure 7 and Table 3 that the time taken for the complete sidekick of all tested athletes varies greatly. Among them, the fastest is still Zhang ^*∗∗*^ of the excellent group, and the overall completion time is 0.864 seconds. The slowest was Qi^*∗∗*^ of the ordinary group, with an overall completion time of 1.153 seconds, a difference of 0.289 seconds between the two. The average duration of complete movement of all athletes was 0.976 ± 0.108 seconds. Knee raising and hip rotation were relatively short, 0.245 ± 0.055 seconds and 0.555 ± 0.064 seconds, respectively. The overall differences among athletes in different groups were very obvious. The phase with the longest time and the greatest difference was the P3 phase, which took 0.802 ± 0.085 seconds. From the above data, it is easy to find that the completion time of elite athletes is generally less than that of ordinary athletes, and the completion time of the overall movement is quite different. The main difference is in the server phase.

#### 4.4.2. Speed Variation Characteristics

With the movement of the human body, the muscles around each joint change from strong to weak from one end close to the limb joint to the farther end. Therefore, according to the size of the cross-sectional area of the muscle, it can be divided into large links and small links. Follow the principle that the big link moves first and drives the small link: when the human body starts to move, it needs to overcome resistance such as gravity. Although the muscles in each link of the kinematic chain will exert force at the same time, the larger link always moves first, driving the nearby small links. The speed of the link with a small mass at the end is also relatively large so the speed of the small link is used to complete the sports technique.

The joint velocity at different times is shown in Figure 8. In the serve phase, the main upper body joint is the wrist. It can be found that at different moments of serving, the change in speed is relatively obvious. Among them, E2 is the fastest, and E4 is the slowest. Among them, since the time E1 is the beginning stage, the initial rate is 0.

#### 4.4.3. The Center of Gravity Changes

As shown in Figure 9, we can obtain the change of the player's center of gravity before and after the server through the video captured by the camera. Among them, the *X*, *Y*, and *Z* directions are illustrated in Figure 5. For different athletes, the change in the center of gravity is not particularly obvious, and the difference between the excellent group and the ordinary group is not very large. This is because, after long-term training, athletes are more aware of their position and will not easily change their center of gravity.

## 5. The Analysis of the Offensive Skills of the Four Volleyball Teams

### 5.1. The Analysis of Serving for the Four Volleyball Teams

As can be seen from Figure 10, in the games of the semifinals: Team L served a total of 139 times in all games, including 0 hooks and 54 frontal overhands, accounting for 38.8%. Vigorously jump serve 85, accounting for 61.2%; team D represents the team in all games, with a total of 125 serves. Among them, there were 0 hooks and 81 frontal overhands, accounting for 64.8%. Vigorously jumped serve 44 times, accounting for 35.2%; Team X has served 136 times in all games. Among them, 17 hooks were served, accounting for 12.5%. Frontal overhand serve 93 times, accounting for 68.4%. 26 times of vigorous jump service accounted for 19.1%; team J has served 107 times in all games. Among them, the hook served 7 times, accounting for 6.5%. Frontal overhand serve 57 times, accounting for 53.2%. Vigorously jumped serve 43 times, accounting for 40.3%.

Among the three serving methods, the hook serve is more aggressive but unstable. The frontal overhand serve is the most stable but less aggressive; the strong jump serve is the most unstable but the most aggressive. In the critical score, most players choose to adjust the hand shape and control strength to reduce the aggressiveness of frontal overhand serve and vigorous jump serve but increase their stability. The hook serve is not easy to control, and the turnover rate is high. Therefore, frontal overhand serve and vigorous jump serve are more suitable for men's volleyball.

### 5.2. Comprehensive Analysis for the Team

In terms of serving methods, the front-handed tap serving is more stable and has fewer mistakes, but the attack is low, and it is easy for the opponent to form an effective attack and score directly. Vigorously, jumping a serve has a greater impact on the opponent's first pass, but the turnover rate is higher. The aggression and stability of the frontal overhand strong serve are at a moderate level compared to the above two serving styles.

In terms of serving effect, the effects of frontal overhand serve and vigorous jump serve have their own advantages and disadvantages. Vigorously, the jumping serve has the highest direct scoring rate and breakage rate, with strong offensiveness and a high turnover rate. The frontal overhand serve has the highest general rate and strong stability, but the direct scoring rate and turnover rate are lower. The hook serve has the highest error rate and the lowest scoring rate, and the effect is poor.

In terms of smashing methods, each team mainly smashes the ball with a strong attack, and the number of fast breaks and tactical attacks is very small. The main reason is that the transmission rate is low and it is difficult to carry out tactical organization. At the same time, the weak awareness of fast break and tactical attack of the offensive players is also an important reason for the single attack method.

In terms of the smashing effect, each team has the best attacking smashing effect, with a higher scoring rate and a relatively stable turnover rate. The fast break is dominated by the No. 3 position. However, due to the intensive blocking of the No. 3 position, the effect is general. In the 2 positions, the “back fast” spiking has a higher direct scoring rate, indicating that there is a large room for improvement in the fast break direction of the No. 2 position and No. 4 position. The tactical offense has the highest direct scoring rate and relatively low turnover rate and is the most effective way to score. However, due to the influence of the first pass and the tactical attack awareness of the attacking players, the number of tactical attacks is less, and the tactics are mostly “echelon” attacks, which are relatively simple.

In terms of lob effect, due to the small field of air volleyball, the lighter weight of the ball, the slower falling speed, and the sufficient time for defenders to move and defend, so the direct scoring rate is low. Most of the scoring situations occur when the thugs go out of bounds by borrowing the blocker. At the same time, lobs that are too close to the net are easily blocked by opponents to score.

In terms of blocking methods, the Jiayuguan team mainly blocks the net with two people, and the Lanzhou Volleyball Association team mainly blocks the net with three people. The Lanzhou City team and the Dingxi City team each accounted for half the proportion of double blocking and three-person blocking. The number of single-person blocks formed by each team is generally less.

In terms of blocking effect, the three-person blocking effect is the best. The main reasons for the failure of the block are the lack of awareness of the blocking players to form three consecutive blocks for multiple rounds, and the slow movement speed of the blocking players. The effect of double blocking is better, but it is easy for opponents to break through and score from outside the blocking range. Solo blocks are concentrated when the setter is close to the net and the attacker cannot make an effective attack. The failure to block the net is mostly due to the insufficient control capability of the blocking hand, causing the thug to go out of bounds.

### 5.3. Advice for Teams

In terms of serving, a serving attack system based on vigorous jump serving should be established. In training, it is necessary to strengthen the aggressiveness of vigorously jumping serves and reduce mistakes. In addition, we should pay attention to the change of the serving line and the landing point to formulate targeted serving tactics according to the receiving position and the characteristics of the first attack of different opponents in the game. At the same time, at least one other form of serving should be proficient. Different ways of serving in the game can affect the opponent's first pass rate to a certain extent.

In terms of spiking, each team should strengthen its ability and awareness to form fast breaks and tactical attacks. According to the characteristics of each team, an effective tactical attack system is formulated, and the net leader can make full use of the opponent's blocking layout to achieve a better offensive effect.

In terms of blocking, it is necessary to take advantage of the short length of the air volleyball net to establish a three-person blocking body. In particular, it is necessary to strengthen the speed of the blocker's movement to the No. 2 position and the ability to form three consecutive blocks for multiple rounds. At the same time, it is necessary to strengthen the training of blocking hands. In addition, when the height of the net is insufficient, the hand shape of the net can be changed to block the net effectively.

Strengthening the training of athletes' psychological quality is the basis for ensuring the use of offensive techniques and offensive effects. It is necessary to cultivate a good style on the court, strengthen the communication between the teams, continue to grow in the game, and ensure that the key games or key scores can be played at their due level.

## 6. Conclusions

Biomechanics is now a more fluid analysis method. It fully references the human body structure. This is a very beneficial way of researching volleyball. This paper firstly explains the related researches on biomechanics and volleyball development and then gives a detailed explanation for the construction of biomechanical models and fully explains volleyball and air volleyball. In the experimental stage, through the image analysis, the relevant indexes of the serving technique were described in detail. Finally, the article analyzes the four strong teams, conducts a more in-depth analysis of the serving technology, and then gives relevant suggestions.

## Figures and Tables

**Figure 1:** Air volleyball.

**Figure 2:** Schematic diagram of a tetrahedral unit.

**Figure 3:** Schematic diagram of hexahedral unit.

**Figure 4:** Schematic diagram of research technology route.

**Figure 5:** Schematic diagram of the experimental test site (top view).

**Figure 6:** Schematic diagram of the stage division of volleyball hitting action.

**Figure 7:** Time characteristics of the two groups of athletes at different stages.

**Figure 8:** Speed of joints at each moment.

**Figure 9:** Changes in the displacement of the center of gravity of the body.

**Figure 10:** Statistics of serving methods.

**Table 1:** Statistical table of testee information.

Sequence	Name	Years	Height	Weight	Set term of years	Group
1	Zhang^*∗*^	23	178	68	8	Excellent group
2	Yang^*∗*^	22	175	66	6	Excellent group
3	Wu^*∗*^	22	173	62	7	Excellent group
4	Zhang^*∗∗*^	24	180	72	10	Excellent group
5	Wang^*∗∗*^	22	165	55	3	Ordinary group
6	Zhao^*∗*^	22	174	72	3	Ordinary group
7	Qi^*∗∗*^	21	170	70	2	Ordinary group
8	Yin^*∗∗*^	22	168	58	3	Ordinary group
Mean		22.25	172.875	65.375	5.25	
Sd		0.829	4.702	6.019	2.727	

**Table 2:** Action stage and action moment table of side kick.

Phase	Event
P1:E1∼E2	E1: Prepare to serve.
P2:E2∼E3	E2: The ball leaves the palm.
P3:E3∼E4	E3: The ball falls back to the palm.
	E4: End of service

**Table 3:** The whole serving time of different athletes.

Athlete	Overall time
Zhang^*∗*^	0.907
Yang^*∗*^	0.885
Wu^*∗*^	0.883
Zhang^*∗∗*^	0.864
Wang^*∗∗*^	0.963
Zhao^*∗*^	1.019
Qi^*∗∗*^	1.153
Yin^*∗∗*^	1.136

## Data Availability

Data sharing is not applicable to this article as no datasets were generated or analyzed during the current study.
